The article "Heterotopic pancreatic cyst in the adrenal gland: A case report and review of literature" was published in 2018. Journal: Medicine (Baltimore).

# Heterotopic pancreatic cyst in the adrenal gland: A case report and review of literature

**DOI:** 10.1097/MD.0000000000009414

**Published:** 2018-01-05

**Authors:** Jianzhong Lin, Yang Yu, Yi Chen, Ming Zheng, Dan Zhou

**Affiliations:** a Department of Urology and Center Laboratory, BenQ Medical Center; b The First Clinical Medical College; c School of Basic Medical Sciences; d Department of Radiology, BenQ Medical Center, Nanjing Medical University, Nanjing, China.

**Keywords:** adrenal gland, cyst, heterotopic, pancreas

## Abstract

**Rationale:**

The incidence of heterotopic pancreas (HP) is relatively rare and mainly found in the upper gastrointestinal tract, and no case of HP cyst in the adrenal gland has been reported. Informed consent has been obtained from the patient for the publication of the case details.

**Patient concerns:**

A 21-year-old woman who presented with chronic lower back pain for a week without urinary disturbance or gastrointestinal discomfortable.

**Diagnoses:**

Ultrasound (US) revealed a left renal cyst, and computed tomography (CT) showed a cyst in the area of the adrenal gland.

**Interventions:**

Cystectomy was successfully performed laparoscopically. Histopathologic examination of the removed cyst wall showed heterotopic pancreatic cyst accompanied by cystic degeneration.

**Outcomes:**

No unusual drainage or abdominal signs were observed during the 6-month follow-up.

**Lessons:**

Despite of its rarity, HP accompanied by cyst formation in the adrenal gland area can present with waist pain. Therefore, the possibility of such disease needs to be considered. For thorough evaluation, in addition to abdominal US, CT, and/or magnetic resonance imaging, histopathological examination should sometimes be performed to make a definite diagnosis. Total excision and regular follow-up is necessary for such cases due to the potential risk of complications or recurrent cyst formation.

## 1 Introduction

Heterotopic pancreas (HP) is a rare congenital anomaly defined as pancreatic tissue that has no contact with the orthotopic pancreas and has its own duct system and vascular supply. It is believed that the pancreatic primordium adhered to original intestine or penetrated the intestinal wall during embryonic development. These primitive bases gradually separated with the changes of the original bowel movement and the pancreas was developed in the gastric, intestinal wall, or mesenteric.^[1]^ Thus, HP can be found in the stomach, duodenum and jejunum, and gallbladder as reported.^[2–4]^ Despite the close anatomic relationship of the adrenal gland and the tail of the pancreas, these 2 organs have different embryologic origins. To date, no case of HP cyst in the adrenal gland has been reported previously. This paper reports the first case of a 21-year-old woman with a cystic formation of the ectopic pancreas in the area of adrenal gland.

## 2 Case report

A 21-year-old woman visited our hospital due to a week of chronic lower back pain without radiation. She had no complaints about urinary disturbances or gastrointestinal discomfort. The pain was not aggravated after excessive meat or alcohol consumption. There was nothing significant about her past personal history and family history.

On physical examination, the patient was well built, her abdomen was soft and nontender, with no palpable mass or percussion pain on either kidney area. The results of routine blood tests and urinalysis were unremarkable. Ultrasound (US) revealed a left renal cyst, and computed tomography (CT) showed a cyst in the adrenal gland area, measuring approximately 5 × 5 cm without reinforcement by contrast-enhanced CT (Figs. 1 and 2). Further detection indicated that blood levels of adrenal hormone (catecholamines, aldosterone, and cortisol) and tumor markers (carbohydrate antigen 19–9 and carcinoembryonic antigen) were within the normal limit. Therefore, she was initially diagnosed as adrenal cyst.

**Figure 1:** Ultrasound revealed a left renal cyst with the size of 5.1 × 4.7 cm.

**Figure 2:** Abdominal computed tomography scan, coronal and sagittal imaging showed the cyst (black arrows), measuring 5 × 5 cm, was located at the superomedial side of kidney closely connected with adrenal gland (white arrows) without abnormal renal morphology. No reinforcement was observed after contrast-enhanced CT scanning.

The cystectomy was successfully performed laparoscopically. The cyst wall was carefully isolated. The volume of postoperative drainage was below 2 mL on the 3rd postoperative day and tube was removed. Histopathologic examination of the removed cyst wall tissue showed cystic degeneration of HP in the left adrenal area (Figs. 3 and 4). She recovered well and was discharged 5 days later and has been remained free of waist pain since then. No cystic structure was found in lesion area with US or CT scan during 6-month follow-up (Figs. 5 and 6).

**Figure 3:** Histological examination of the resected specimen showed lobules of the pancreatic tissue with acini (black triangle), ducts (white arrow), islets (white triangle), and cystic area (black arrow) was coated with cuboidal epithelial tissue (H&E, ×100). H&E = hematoxylin-eosin staining.

**Figure 4:** Histological examination of the resected specimen showed features of abnormal pancreatic islets (black arrows) and ducts (white arrow) was adjacent to a small part of the adrenal tissue (black triangle) (H&E, ×40, ×200).

**Figure 5:** Ultrasound demonstrated the normal shape of adrenal gland (white arrow), kidney and pancreas. The cyst disappeared after surgery.

**Figure 6:** Computed tomography revealed no cystic structure in lesion area, with a relatively normal morphology of adrenal gland (white arrow) and pancreas (black arrows).

## 3 Discussion

HP has a genetic alteration, physiologic function, and local environmental exposure similar to that of the pancreas. It is often an incidental finding, with a reported incidence of approximately 0.2% at laparotomy and 13.0% at autopsy, and most commonly found in the stomach (25%–38%), duodenum (17%–21%), and proximal jejunum (15%–21%).^[5,6]^ HP is usually asymptomatic and found during imaging, endoscopy, or upper abdominal operations, but may become clinically evident depending on its size and the pathological changes (cyst formation, pancreatitis, and malignant degeneration). Most ectopic pancreases measure less than 2 cm in size and the diagnosis of HP is difficult as there are no specific diagnostic methods, leading to be misdiagnosed preoperatively in most of the patient.^[7]^

In this case, US showed a left renal cyst, CT, coronal and sagittal imaging demonstrated the cyst was located at the superomedial side of kidney, closely connected with adrenal gland without abnormal renal morphology. Some research reports have reported that pheochromocytoma or neoplasm can present as adrenal cystic lesion.^[8,9]^ Therefore, the levels detection of hormone secreted by adrenal glands and enhanced CT scanning was performed accordingly. The normal hormone levels and no reinforcement effect were observed. A diagnosis of adrenal cyst was preliminarily made based on the clinical presentations and imaging. The cyst with a diameter of 5 cm has made the patient feel pain at waist and was then treated by retroperitoneoscopic.

Surprisingly, HP accompanied by cyst formation was confirmed by pathology in this case and possessed acini, duct, and islets similar to those seen in normal pancreas. Furthermore, the typical surface epithelium of pancreas cyst was found and indicated the cyst should be congenital, in contrast to the walls of pancreatic pseudocyst, which do not contain epithelial components. True cysts are commonly classified into congenital–developmental cysts, retention cysts, or duplication cysts. It is accepted that true cysts occur as a result of developmental anomalies related to the sequestration of primitive pancreatic ducts.^[10]^ In this case, the presence of abnormal pancreatic ducts, in addition to the epithelial component on the cystic wall, was further indicative of a congenital heterotopic true pancreatic cyst.

In congenital cystic fluid, low enzymatic activity is generally observed, whereas enzymatic activity of retention cysts is considerably high.^[11]^ Enzymatic activity detection of cystic fluid of this patient was not carried out since we considered the cyst origin from adrenal gland before the pathological result. Fortunately, complete resection and adequate drainage were performed for this patient and the recovery was successful without complications caused by trypsin. If the detection was examined, it would be helpful for understanding the exact cause of this true cyst.

At present, surgical resection should be performed if HP is symptomatic or when the lesion is larger than 3 cm in size, in order to prevent complications.^[12,13]^ Laparoscopic surgery is thought to be technically feasible and safe. In this case, since the cyst is large and adjacent to pancreas, careful isolation was performed to avoid pancreatic injury. The cyst was completely resected with a small part of adrenal gland removed for obvious adhesion between them, which was further confirmed by pathology (Fig. 4). There were no unusual drainage or abdominal signs after surgery. In terms of the patient, it can be assumed that her pancreas was fully protected based on postoperative recovery and imaging follow-up.

Malignant transformation of HP has been reported, although it is difficult to determine its true incidence.^[14,15]^ Postoperative follow-up is necessary for these patients. In our case, no similar pain occurred in the patient's left waist again after discharge. US and CT scan showed no cystic structure in lesion area during 6-month follow-up.

In conclusion, despite of its rarity, HP accompanied by cyst formation in the adrenal gland area can present with waist pain. Therefore, the possibility of such disease needs to be considered. Thorough evaluation, abdominal US, CT, and/or magnetic resonance imaging should be performed. Intraoperative biopsy may sometimes be considered and total excision with such cyst is preferred to avoid some complications. Regular follow-up is necessary due to the potential risk of recurrent cyst formation and malignant transformation.
